# Inverse Relationship of the* CMKLR1* Relative Expression and Chemerin Serum Levels in Obesity with Dysmetabolic Phenotype and Insulin Resistance

**DOI:** 10.1155/2016/3085390

**Published:** 2016-04-28

**Authors:** Fernanda-Isadora Corona-Meraz, Rosa-Elena Navarro-Hernández, Sandra-Luz Ruíz-Quezada, Perla-Monserrat Madrigal-Ruíz, Jorge Castro-Albarrán, Efraín Chavarría-Ávila, Milton-Omar Guzmán-Ornelas, Eduardo Gómez-Bañuelos, Marcelo-Herón Petri, Joel-Isidro Ramírez-Cedano, María-Elena Aguilar-Aldrete, Clara Ríos-Ibarra, Mónica Vázquez-Del Mercado

**Affiliations:** ^1^Departamento de Biología Molecular y Genómica, Centro Universitario de Ciencias de la Salud, Universidad de Guadalajara, Sierra Mojada No. 950 Colonia Independencia, CP 44340, Guadalajara, JAL, Mexico; ^2^Instituto de Investigación en Reumatología y del Sistema Musculo Esquelético, Centro Universitario de Ciencias de la Salud, Universidad de Guadalajara, Sierra Mojada No. 950 Colonia Independencia, CP 44340, Guadalajara, JAL, Mexico; ^3^UDG-CA-701, Grupo de Investigación Inmunometabolismo en Enfermedades Emergentes (GIIEE), Centro Universitario de Ciencias de la Salud, Universidad de Guadalajara, Sierra Mojada No. 950 Colonia Independencia, CP 44340, Guadalajara, JAL, Mexico; ^4^Departamento de Farmacobiología, Centro Universitario de Ciencias Exactas e Ingenierías, Universidad de Guadalajara, Boulevard Marcelino García Barragán No. 1421, CP 44430, Guadalajara, JAL, Mexico; ^5^Departamento de Disciplinas Filosófico, Metodológico e Instrumentales, Centro Universitario de Ciencias de la Salud, Universidad de Guadalajara, Sierra Mojada No. 950 Colonia Independencia, CP 44340, Guadalajara, JAL, Mexico; ^6^UDG-CA-703, Grupo de Investigación en Inmunología y Reumatología, Centro Universitario de Ciencias de la Salud, Universidad de Guadalajara, Sierra Mojada No. 950 Colonia Independencia, CP 44340, Guadalajara, JAL, Mexico; ^7^Translational Cardiology, Centre for Molecular Medicine, Department of Medicine, Karolinska Institutet, L8:03, 17176 Stockholm, Sweden; ^8^Servicio de Reumatología, División de Medicina Interna, Hospital Civil “Dr. Juan I. Menchaca”, Universidad de Guadalajara, Salvador de Quevedo y Zubieta No. 750, CP 44340, Guadalajara, JAL, Mexico

## Abstract

*Background*. In obesity there is a subclinical chronic low-grade inflammatory response where insulin resistance (IR) may develop. Chemerin is secreted in white adipose tissue and promotes low-grade inflammatory process, where it expressed* CMKLR1* receptor. The role of chemerin and* CMKLR1* in inflammatory process secondary to obesity is not defined yet.* Methods*. Cross-sectional study with 134 individuals classified as with and without obesity by body mass index (BMI) and IR. Body fat storage measurements and metabolic and inflammatory markers were measured by routine methods. Soluble chemerin and basal levels of insulin by ELISA and relative expression of* CMKLR1 *were evaluated with qPCR and 2^−ΔΔC_T_^ method.* Results*. Differences (*P* < 0.05) were observed between obesity and lean individuals in body fat storage measurements and metabolic-inflammatory markers. Both* CMKLR1* expression and chemerin levels were increased in obesity without IR. Soluble chemerin levels correlate with adiposity and metabolic markers (*r* = 8.8% to 38.5%), *P* < 0.05.* Conclusion*. The increment of* CMKLR1 *expression was associated with insulin production. Increased serum levels of chemerin in obesity were observed, favoring a dysmetabolic response. The results observed in this study suggest that both chemerin and* CMKLR1* have opposite expression in the context of low-grade inflammatory response manifested in the development of IR.

## 1. Introduction

Obesity which is the excess storage of white adipose tissue (WAT) and low-grade inflammation are the key factors for development of insulin resistance (IR) [1–4].

In WAT primed immune cells are recruited as adiposity increases, and these cells became resident cells (mainly macrophages) and secrete proinflammatory adipokines that promote further recruitment of circulating monocytes [4–7]. Later, they polarize towards M1 macrophages, favoring an inflammatory subclinical chronic state [6, 8–10].

Chemerin is an adipokine secreted by adipocytes; it is closely associated with amount of fat and distribution. As a chemoattractant protein, chemerin acts as a ligand for the coupled G-receptor protein (ChemR23) and participates in both adaptive and innate immunity [11]. In humans, chemerin gene (*RRARES2*) is highly expressed in WAT and to a lesser extent in liver and lungs. On immune cells, chemerin is known to stimulate chemotaxis of dendritic cells, macrophages, and NK cells. Meanwhile, its receptor, ChemR23 gene (*CMKLR1*), is expressed in dendritic cells, monocyte/macrophages, and endothelial cells [11–14]. ChemR23 is involved in the differentiation of adipocytes and increased intracellular glucose or lipids promote its expression [14].

The interaction of chemerin/ChemR23 has been shown to reduce cytokines, chemokines, and phagocytosis, proving to be important in the inflammatory process associated with obesity [12, 14, 15].

In this context, chemerin/ChemR23 axis has been shown to impact IR development, which influences the clinical course and severity of obesity-related diseases [10]. However, the association with immunometabolic markers and chemerin and its receptor ChemR23 is scarce. Therefore, the aim of this study was to characterize the inflammatory and metabolic phenotype of subjects with obesity-IR state based on the chemerin soluble levels and its receptor* CMKLR1* expression.

## 2. Material and Methods

### 2.1. Study Design

In this cross-sectional study a total of 134 adults, aged 20 to 59 years, were recruited from general population in the west of Mexico. We included individuals who at the time of enrollment did not present glucose intolerance, infectious diseases, hypertension, pregnancy, anemia, cardiovascular disease, malignancy, and renal and metabolic diseases such as type 2 diabetes mellitus (T2DM). Subjects with current medication use were excluded.

Subjects were classified in two forms, based on obesity and then by IR. First, they were classified according to the recommendations' of World Health Organization, by body mass index (BMI), waist circumference (WC), waist-hip ratio (WHR), and waist to height ratio (WHtR), in two groups: subjects with obesity, if any of the following conditions were present: BMI ≥ 30.0 kg/m^2^, WC ≥ 90.0 cm, WHR ≥ 0.90, and WHtR ≥ 52.5 in Men and WC ≥ 80.0 cm, WHR ≥ 0.80, and WHtR ≥ 53.0 in women, and lean subjects that are lower in these measurements. For detection of IR in subjects with obesity they were secondly classified according to Gayoso criteria in two groups: with and without IR [16].

For ethical purposes, participants were informed about the study and signed a consent form following the Helsinki declaration guidelines [17] and the institutional (Guadalajara University) review boards' committees.

### 2.2. Subjects' Medical History and Physical Examination

All individuals who satisfied inclusion criteria were clinically evaluated by a physician who performed a complete medical history. Assessment of general health status and vital signs were included: blood pressure (measured 3 times with the subject in the sitting position for 15 minutes before the evaluation), heart and respiratory rate, and body temperature.

### 2.3. Subjects' Body Fat Storage Measurements

We evaluated height, which was measured to the nearest 1 mm by using a stadiometer (Seca GmbH & Co. KG. Hamburg, Germany); body weight and total and trunk body fat mass (absolute, kg, and relative, %) were determined by bioelectrical impedance analysis (TANITA BC-418 Segmental Body Composition Analyzer, Tokyo, JPN) to the nearest 0.1 kg. WC, hip circumference (HC), and coronal abdominal diameter were measured by using an anthropometric fiberglass tape (GULICK® length 0–180 cm precision ±0.1; USA). At the level of the iliac crest (L4-5) sagittal abdominal diameter was measured using a sliding-beam, abdominal caliper (precision ±0.1 cm, Holtain Ltd. Crosswell, Crymych, Pembs., SA41 3UF, UK) with the patient lying in a supine position on the examination table [18]. Five measures of skinfold thickness (i.e., abdominal, bicipital, tricipital, subscapular, and suprailiac) were obtained on the right side of the body by using a Harpenden skinfold caliper (opened 80 mm with precision of ±0.2 mm, constant pressure: 10 g/mm^2^; Holtain Ltd. Crosswell, Crymych, Pembs., SA41 3UF, UK). All these measurements were carried out by the same Physician, in duplicate following the procedures recommended by anthropometric indicators measurement guide [19, 20].

To determine obesity and adiposity indexes the following calculations were used: BMI, kg/m^2^ = weight (kg)/height^2^ (m); WHtR = WC (cm)/height (cm) [21]; WHR = WC (cm)/HC (cm); conicity index (CI) = WC (cm)/$0.109\sqrt{\left(weight\;(kg)/height\;(cm)\right)}$; BFR = total body fat mass (kg)/height (cm); total adipose area (TAA, cm^2^) = WC^2^/4*π*; visceral area (VA, cm^2^) = *π*(WC/2*π*  −  abdominal skinfold)^2^; subcutaneous abdominal area (cm^2^) = TAA − VA [18]; visceral adiposity index (VAI): for males, VAI = (WC/36.58 + (1.896BMI))6(TG/0.81)6(1.52/HDLc) and females, VAI = (WC/39.68 + (1.886BMI)) 6(TG/1.03)6(1.31/HDLc) [22]; homeostasis model assessment-insulin resistance (HOMA-IR) = [basal glucose mg/dL × (basal insulin *μ*UI/mL)/405] [23, 24].

### 2.4. Metabolic, Inflammatory Markers, and Chemerin Levels Measurements

Individuals included in the study were fasting 12 hours before the blood samples were taken, allowing them to clot at room temperature, and then were centrifuged at 1509 RCF (Rotanta 460R, Andreas Hettich GmbH & Co. KG.) for 10 minutes at 20°C. Serum was collected and stored at −86°C until further analysis.

We quantified serum concentration of glucose and nonesterified fatty acids (NEFA) with routine enzymatic methods; triglycerides (TG) and total cholesterol (TC) with routine colorimetric methods, high and low density lipoprotein cholesterol (HDLc and LDLc, resp.), apolipoproteins A1 (Apo-A1) and B (Apo-B), and high sensitivity C reactive protein (CRP) with immunoturbidimetry methods (Randox Laboratories 55 Diamond Road, Crumlin Co. Antrim, Northern Ireland, UK); and erythrocyte sedimentation rate (ESR) with Wintrobe method [25]. And the low density lipoprotein cholesterol (VLDLc) was obtained with the Friedewald formula [26].

Through using commercial enzyme-linked immunoabsorbent assays (ELISA) soluble levels of insulin were determined (sensitivity of 0.399 *μ*UI/mL) (ALPCO 26-G Keewaydin Drive, Salem, NH 03079), and chemerin was determined with a limit of detection of 1.08–7.8 ng/mL (R&D Systems, Minneapolis, USA).

### 2.5. CMKLR1 Relative Expression Analysis

Mononuclear cells from the subjects studied were isolated by density gradient media with separating solution Lymphoprep*™* (AXIS-SHIELD PO Box  6863 Rodelokka, 0504 Oslo, Norway). Total RNA was isolated from purified mononuclear cells, using TRIzol® LS Reagent (Ambion RNA Life Technologies, 5791 Van Allen Way, Carlsbad, CA 92008) based on the single-step RNA isolation modified method reported by Chomczynski [27]. Complementary DNA synthesis (cDNA) was performed with 2 *μ*g of each total RNA sample using a reaction size of 20 *μ*L, with oligo (dT) 18 primer (100 ng/*μ*L), RNase free, DEPC treated water, and SuperScript Reverse Transcriptase III kit (Applied Biosystems, 850 Lincoln Centre Drive, Foster City, CA 94404) and stored at −20°C until used for expression analyses.

Real-Time Quantitative Polymerase Chain Reaction (qPCR) was conducted using the StepOne*™* detection system, EXPRESS SYBR® GreenER*™*, and ROX*™* qPCR SuperMix Universal, and sequence detector software v2.3 (Applied Biosystems, 850 Lincoln Centre Drive, Foster City, CA 94404) was used for data analysis. A threshold cycle (CT) value was determined from each amplification plot.

In brief,* CMKLR1* mRNA expression was performed in a final reaction volume of 20 *μ*L (10 *μ*M forward and reverse primer, 500 nM ROX, 1X SYBR Green qPCR master mix, and cDNA 1000 ng). The conditions of the reaction were as follows: holding 95°C/10 min, cycling (35 cycles of 95°C/15 s, 60°C/60 s), and melt curves 95°C/15 s, 60°C/60 s, and 95°C/15 s. Expression of target genes was normalized by the endogenous reference gen* RPS28*; sequence specific primers were forward: 5′-GGTCTGTCACAGTCTGCTCC-3′, and reverse 5′-CATCTCAGTTACGTGTGGCG-3′ and for* CMKLR1* target gen forward: 5′-GTGGTGGTCTACAGCATCGT-3′ and reverse: 5′-ATGGCGGCATAGGTGATATGG-3′.

The relative expression fold change of target gene was calculated using the comparative CT method with 2^−ΔΔC_T_^ equation [28]. To ensure accuracy of data, experiments were done in duplicate, blank, internal controls and melt curve data were collected with applications of StepOne detector software (Cat. 4376357).

### 2.6. Statistical Analysis

Data were analyzed with statistics software SPSS v21 (IBM Inc., Chicago, IL, USA) and GraphPad Prism v6.01 (2014 Inc. 2236 Beach Avenue Jolla, CA 92037). Results are given as mean ± standard deviation (SD). The data distribution of clinical and laboratory variables was evaluated with *Z* Kolmogorov-Smirnov test. The clinical and laboratory characteristics of study group were compared with one way ANOVA with Tukey* post hoc*. Data from serum concentrations of chemerin and insulin, laboratorial assessment, and adiposity variables were subjected to Pearson correlation tests. A two-tailed *P* value < 0.05 was considered statistically significant.

## 3. Results

### 3.1. Status Assessment of Body Fat Showed High Adiposity and IR

In this study, the observed frequency of obesity and IR was 63% and 39%, respectively, while IR was not present in lean individuals (with average BMI of 21.6 kg/m^2^, 18.0 to 24.7). For individuals classified with obesity, IR prevalence was 62%. The adiposity measurements are shown in Table 1.

The fat distribution assessed by the skinfold thicknesses showed magnitudes as follows: the group with obesity and IR > obesity without IR group > lean group (Figure 1(a)). Adiposity indexes were increased in both groups with obesity* versus* lean subjects, except VAI whose increase is observed in individuals with IR* versus *lean subjects (Figure 1(b)).

### 3.2. Individuals with Obesity and IR Presented a Subclinical Inflammatory State and Dyslipidemia

Lean individuals presented lower levels of glucose, insulin, and HOMA-IR when compared with individuals with and without IR, whereas NEFA presented no changes in different groups (Figure 1(c)); lean individuals showed lower levels of triglycerides and LDLc compared to subjects with and without IR, also lean individuals presented lower levels of total cholesterol and VLDLc when compared to obesity group with IR. Lean subjects also presented lower levels of Apo-B compared with individuals without IR whereas HDLc and Apo-A1 presented no statistical changes (Figure 1(d)). Levels of CRP and ESR were higher in obesity with IR* versus* lean (6.83 ± 5.65, 17.46 ± 11.67, *P* < 0.001; resp.).

### 3.3. Obesity without IR Showed a Contrasting Context on Chemerin Levels

Increased levels of soluble chemerin were observed in obese individuals without IR compared to obese individuals with IR and lean subjects groups (Figure 2(a)).

### 3.4. Chemerin and Insulin Levels Were Associated with Dysmetabolic Phenotype and Body Fat Adiposity Markers

Positive correlations of chemerin and insulin were observed with the increase in the status of body fat and subcutaneous fat accumulation with lipid profile (Table 2).

### 3.5. Higher* CMKLR1* Relative Expression Was Associated with Obesity without IR

Increased expression levels of* CMKLR1 *receptor were observed in individuals with obesity without IR* versus* lean and obesity with IR individuals (Figure 2(b)).

A detailed test by tertiles was performed (describing the first tertile as lower expression, second tertile as intermediate expression, and third tertile as higher expression); we found increased accumulation of abdominal fat mass and metabolic markers between individuals with high expression* versus* individuals with low expression of* CMKLR1*, independent of the presence of IR and/or obesity. Other relevant information provided in this analysis is that there is an inverse correspondence in insulin levels, HOMA-IR, and NEFA regarding the expression of* CMKLR1* (Table 3).

## 4. Discussion

Two main findings emerge from this study: first, the* CMKLR1 *receptor expression was associated with obesity and its features, and second, its ligand chemerin was associated not only with obesity, but also with metabolic dysfunction such as dyslipidemia and IR.

Adipose tissue has been suggested to be an important source of low-grade inflammation based on three biological aspects: quantity (total mass and relative proportion), anatomical distribution, and phenotype of resident cells [10, 29].

Regarding the quantity and site, our study supported that dysfunctional WAT may play an important role in low-grade inflammation, because the individuals with obesity shown increased accumulation of fat manly in the abdominal region along with low-grade inflammation and dysmetabolic phenotype (represented by dyslipidemic state and increased adiposity indexes), although not all individuals with obesity were IR.

Another important point from this study is that it supports the fact that the IR is a component for developing a chronic-degenerative disease. The IR first promotes dyslipidemia (as an intermediate event) leading to metabolic syndrome and subsequently development of T2DM [1, 3, 30].

The dysmetabolic phenotype observed in individuals with obesity in our study can be explained in the context of immune system dysregulation that exists in IR by the development of two alternative mechanisms not exclusive: in one the WAT of individuals with obesity have increased resident M1 macrophages able to produce chemokines and in additional one, it has been found that high concentrations of fatty acids induce expression of TNF*α* and Toll-like receptor-4 signaling [4, 30]. This pathway converges with insulin signaling in adipocytes affecting positively glucose transport, glycogen synthesis, and cell differentiation while negatively affecting the lipolysis and gluconeogenesis [8, 31, 32].

The polarization of monocytes/macrophages to M1 in WAT is favored by coupling of chemerin through ChemR23 that in turn displayed a proinflammatory profile, where chemotactic ligand-receptor interaction regulates continued migration of monocytes to WAT [13, 14]. Soluble chemerin produced by adipocytes and resident macrophages M1 in WAT binds to ChemR23 with high affinity, and its levels decrease as recruited circulating monocytes differentiate into macrophages [12–14, 33, 34].

This study evaluated the gene expression of* CMKLR1* receptor in circulating monocytes. It presented 7.9- or 3.8-fold higher expression in individuals with obesity without IR or obesity with IR, respectively, than lean individuals. Interestingly the increase in expression levels was directly associated with the proportion of abdominal fat mass and body dimensions, whereas an inverse association was observed with the production of insulin, nonesterified free fatty acids, and HOMA-IR.

In this regard, previous study showed that the chemerin/ChemR23 signaling does not affect the inflammatory response in* ex vivo* human macrophages [35]. The expression levels of* CMKLR1* found in our study suggest that the level of expression is higher in early activation of primed circulating monocytes but decreases at later stages, which can be explained based on the reports in other studies in animal models [31, 36], although changes of* CMKLR1* expression in human macrophage differentiation/polarization still remain to be established.

The association of* CMKLR1* expression levels, observed in our study, can be explained due to IR being closely associated with excess in abdominal accumulation of WAT [30] and based on other reports in which an adipocyte cell line expression of* CMKLR1* was analyzed during differentiation process where upregulation was in the early stage whereas a downregulation was observed in late stages [37, 38]. Proinflammatory stimulus such as TNF*α* or adiponectin has been shown to upregulate gene expression of* CMKLR1* in differentiated adipocytes [39]. This shows the complexity of the* CMKLR1* expression and functionality that is not dependent on the expression of its ligand but also dependent on the cell type presented on the disease.

Nevertheless, the limitations of this study were that protein levels of the ChemR23 in monocyte were not assessed, limiting complementary studies about the functional receptor. Another limitation that should be taken in consideration is that this same receptor is known to bind with the same affinity to the lipid mediator resolving E1, which has anti-inflammatory properties. The quantification of such ligand was not done.

One of the main findings was the increased serum levels of chemerin in individuals with obesity without IR* versus* individuals with IR and lean. In parallel correlation with indicators of adiposity and metabolic markers was observed.

In this regard, previous studies report conflicting results on chemerin levels in different diseases with an inflammatory component such as chronic pancreatitis (94.0 ng/mL) [40], T2DM individuals (179.0 ng/mL) [41], lipodystrophy (234.3 ng/mL) [42], and obesity without diabetes (590.08 ng/mL) [43]. Chemerin levels were increased, except for the levels reported in rheumatoid arthritis (35.0 ng/mL) [44] (an inflammatory disease* per se*), although this can be explained based on treatment; however, other studies have suggested that chemerin may be the functional link between chronic inflammation and obesity-related T2DM and cardiovascular disease [45].

Our results can be explained because monocytes/macrophages are decisive in the pathogenic process of IR, based on the fact that they are an important source of proinflammatory markers (TNF*α*, IL-6, chemerin, and C reactive protein), along with increased levels of expression of adipokines, chemokines, and proinflammatory cytokines associated with an equivalent increase in hyperplastic and hypertrophic adipocytes [13, 30, 46].

One important observation from this study is that, in the context of obesity, soluble chemerin levels enhanced both the inflammation and dysmetabolic phenotype, showing how an opposite change in the expression of* CMKLR1* takes place once IR is established.

In previous reports it is postulated that chemerin production has a dual profile pro/anti-inflammatory [9, 15]. In this context we suggest that, in the initial stage of IR, the increase in chemerin levels promotes dysmetabolic profile arising from the dysfunctional adipose tissue [36]. Although in the setting of obesity during the process of establishment of IR the levels of chemerin can be decreased, the dysmetabolic profile is maintained. Its scenery might be explained due to that action of chemerin where it regulates the insulin metabolism [6].

## 5. Conclusions

This is the first study that links the increment of* CMKLR1 *expression with insulin production, showing an association with fat mass and corporal dimensions, while the increased serum levels of chemerin in obesity were observed, favoring a dysmetabolic response.

Taking together, the results observed in this study suggest that both chemerin and* CMKLR1* have opposite expression in the context of low-grade inflammatory response, manifested in the development of IR.

Functional studies are necessary to clarify the biological functions of chemerin signaling in the pathogenesis of IR.

## Figures and Tables

**Figure 1:** Body fat mass distribution, adiposity indexes, and metabolic markers in the study groups. Lean: [BMI: 21.4 (18.5–24.7) kg/m^2^] *n* = 49; obesity without IR: [BMI: 32.0 (30.1–34.7) kg/m^2^] *n* = 32; obesity with IR: [BMI: 32.6 (30.2–34.9) kg/m^2^] *n* = 53. IR: insulin resistance. WHtR: waist to height ratio; WHR waist-hip ratio; CI: conicity index; VAI: visceral adiposity index; BFR: body fat ratio; HOMA-IR: homeostatic model assessment of insulin resistance; NEFA: none esterified fatty acids; TG: triglycerides; TC: total cholesterol; HDLc, LDLc, and VLDLc (lipoproteins of high, low, and very low density cholesterol, resp.). Data are shown in $\overset{-}{x}\pm SD$. ^*∗∗*^ *P* < 0.001, ^*∗*^ *P* < 0.05 (ANOVA, Tukey* post hoc*).

**Figure 2:** Levels of soluble chemerin and relative expression of* CMKLR1* in the study groups. (a) Relative expression of* CMKLR1*. Method 2^−ΔΔC_T_^: ^*∗*^difference between obesity without IR and lean (7.9-fold; *P* = 0.003), and ^*∗∗*^obesity with IR* versus* lean (3.8-fold; *P* < 0.001). (b) Serum levels of chemerin (ANOVA, Tukey* post hoc*). IR: insulin resistance.

**Table 1:** Status of body fat storage in individuals in the study group.

Study group	Lean	Obesity without IR	Obesity with IR
BMI (kg/m^2^)	[21.6 (18.5–24.7)]	[32.0 (30.1–34.7)]	[32.6 (30.2–34.9)]
*n* = 134	49	32	53

*Measurement*			
Height (cm)	166.0 ± 8.4	162.8 ± 7.8	163.8 ± 9.0
Body weight (kg)	60.0 ± 9.9	90.1 ± 12.8^a^	97.3 ± 18.9^a^
Total body fat mass (%)	20.3 ± 5.9	40.3 ± 6.8^a^	40.6 ± 6.9^a^
Total body fat mass (kg)	12.0 ± 3.6	36.6 ± 8.8^a^	39.8 ± 12.4^a^
Trunk body fat mass (%)	23.8 ± 10.6	38.1 ± 11.4^a^	35.4 ± 10.5^a^
Trunk body fat mass (kg)	5.9 ± 2.4^b,c^	18.4 ± 3.9^a,c^	19.4 ± 6.1^a,b^
Waist circumference (cm)	78.3 ± 6.6	109.6 ± 11.9^a^	113.7 ± 13.2^a^
Hip circumference (cm)	93.3 ± 4.8	115.7 ± 12.4^a^	118.8 ± 10.8^a^
Coronal abdominal diameter (cm)	30.2 ± 6.4^b,c^	38.0 ± 8.7^a,c^	44.9 ± 12.0^a,b^
Sagittal abdominal diameter (cm)	16.7 ± 2.1	24.6 ± 3.4^a^	25.9 ± 4.4^a^
Total adipose area (cm^2^)	491.2 ± 82.3	967.9 ± 216.6^a^	1042.5 ± 249.6^a^
Visceral area (cm^2^)	227.4 ± 373.0	292.7 ± 516.4	599.7 ± 836.1^a^
Subcutaneous abdominal area (cm^2^)	314.2 ± 324.0	696.8 ± 560.8^a^	562.6 ± 908.7

BMI: body mass index [$\bar{x}$ (min–max)]. Data are shown in $\bar{x}$  ± SD. ^a^Difference *versus* lean. ^b^Difference *versus* obesity without IR. ^c^Difference *versus* obesity with IR (*P* < 0.05, ANOVA, Tukey *post hoc*). IR: insulin resistance.

**Table 2:** Correlation of chemerin and insulin serum levels with the dysmetabolic phenotype and body fat adiposity markers status in the study groups.

Measurements	Chemerin (ng/mL)	Insulin (*μ*UI/mL)
	Correlation (%)	
Body weight (kg)	−2.8	34.7^**∗∗**^
BMI (kg/m^2^)	15.3	46.2^**∗∗**^
Body fat mass (%)	38.5^**∗∗**^	41.5^**∗∗**^
Total body fat mass (kg)	26.1^**∗∗**^	46.7^**∗∗**^
Waist circumference (cm)	18.8^**∗**^	36.4^**∗∗**^
Hip circumference (cm)	21.6^**∗∗**^	41.5^**∗∗**^
Waist-hip ratio	5.8	16.9^**∗∗**^
Body fat ratio	31.5^**∗∗**^	47.1^**∗∗**^
Waist to height ratio	26.6^**∗∗**^	38.8^**∗∗**^
Conicity index	30.7^**∗∗**^	18.3^**∗∗**^
Coronal abdominal diameter (cm)	8.4	13.0^**∗**^
Sagittal abdominal diameter (cm)	15.7	46.4^**∗∗**^
Total adipose area (cm^2^)	18.8^**∗**^	36.4^**∗∗**^
Visceral area (cm^2^)	19.2^**∗**^	37.0^**∗∗**^
Subcutaneous abdominal area (cm^2^)	17.6	19.4^**∗∗**^
Glucose (mg/dL)	−6.3	22.5^**∗∗**^
Skinfold thickness (mm):		
Abdominal	−10.3	17.3^**∗∗**^
Bicipital	32.7^**∗∗**^	45.8^**∗∗**^
Tricipital	30.4^**∗∗**^	39.0^**∗∗**^
Subscapular	11.1	38.8^**∗∗**^
Suprailiac	16.1^**∗**^	36.5^**∗∗**^
Triglycerides (mg/dL)	20.4^**∗**^	26.1^**∗∗**^
LDLc (mg/dL)	13.0	12.5^**∗**^
VLDLc (mg/dL)	20.4^**∗**^	20.9^**∗∗**^
HDLc (mg/dL)	17.4^**∗**^	10.1
NEFA (mmol/L)	30.2^**∗∗**^	9.0
CRP (mg/L)	14.1	31.5^**∗∗**^
ESR (mm/h)	30.2^**∗∗**^	1.8

IR: insulin resistance. HDLc, LDLc, and VLDLc (lipoproteins of high, low, and very low density cholesterol, resp.); NEFA: nonesterified fatty acids; CRP: C reactive protein; ESR: erythrocyte sedimentation rate. ^**∗∗**^ *P* < 0.001, ^**∗**^ *P* < 0.05, Pearson correlation test.

**Table 3:** Adiposity and metabolic markers in the relative expression levels of *CMKLR1.*

Tertile	First	Second	Third
*CMKLR1 *relative expression	[0.546 (0.034–1.060)]	[4.148 (1.148–8.934)]	[69.787 (9.009–473.260)]
% obesity	48.7	44.1	51.7
% IR	59.0	52.9	48.3

*Measurement*			
Trunk body fat mass (%)	26.02 ± 12.0	32.32 ± 9.0^a^	33.37 ± 6.4^a^
Coronal abdominal diameter	35.15 ± 12.0	42.18 ± 10.5^a^	40.97 ± 8.9
VAI	2.44 ± 2.6	3.33 ± 2.3	4.54 ± 2.41^a^
Insulin (*μ*UI/mL)	15.22 ± 11.4	13.08 ± 8.4	8.74 ± 5.1^a^
HOMA-IR	3.49 ± 2.5	3.05 ± 1.9	2.13 ± 1.4^a^
NEFA	0.725 ± 0.2	0.618 ± 0.26	0.500 ± 0.25^a^

The expression levels of *CMKLR1* are in relative units [$\bar{x}$ (min–max)]. Data are shown in $\bar{x}$  ± SD and were classified by tertiles. ^a^Difference *versus* first tertile (*P* < 0.05, ANOVA, Tukey *post hoc*). IR: insulin resistance. VAI: visceral adiposity index; HOMA-IR: homeostatic model assessment of insulin resistance; NEFA: nonesterified fatty acids.
